# Vomiting Management and Effect Prediction after Early Chemotherapy of Lung Cancer with Diffusion-Weighted Imaging under Artificial Intelligence Algorithm and Comfort Care Intervention

**DOI:** 10.1155/2022/1056910

**Published:** 2022-06-15

**Authors:** Cailing Mei, Ling Zhang, Zhiying Zhang

**Affiliations:** ^1^Department of Oncology, Ganzhou People's Hospital, Ganzhou, 341000 Jiangxi, China; ^2^Department of Nursing, Ganzhou People's Hospital, Ganzhou, 341000 Jiangxi, China; ^3^Department of Medical Imaging, Ganzhou People's Hospital, Ganzhou, 341000 Jiangxi, China

## Abstract

This aim of this research was to explore the evaluation and prediction value of diffusion-weighted imaging (DWI) under artificial intelligence algorithm in the vomiting management and chemotherapy of early lung cancer under comfort care. 118 patients with lung cancer were included as the research objects. They were randomly divided into the control group (routine care) and the experiment group (comfort care) with 59 cases in each. The DWI under the weighted nuclear norm minimization (WNNM) noise reduction algorithm was used for examinations. The noise reduction effect of the algorithm under different Gaussian noises, as well as the sensitivity, specificity, and area under the curve (AUC) of the apparent diffusion coefficient (ADC) maps under different *b* values, was compared and analyzed. The indicators of vomiting, psychological state, quality of life, serum tumor marker levels, and nursing satisfaction were also compared between the two groups of patients after chemotherapy. Compared to the photon mapping (PM) algorithm and the total variation (TV) norm minimization algorithm, the WNNM algorithm had the most ideal noise reduction effect with clearer images, which was conducive to identification. When the *b* value was 800 s/mm^2^, the ADC chart had the best sensitivity, specificity, and AUC values of 0.95, 0.89, and 0.87, respectively. After chemotherapy, 45.76% of patients in the experiment group had vomiting in degree 0 and 40.68% had that in degree I, which suggested that the incidence of vomiting was significantly lower than that in the control group (*P* < 0.05). All of the psychological state, quality of life, serum tumor marker levels, and nursing satisfaction of patients in the experiment group were significantly better than those in the control group (*P* < 0.05). It showed that comfort care could alleviate the vomiting response effectively of patients with lung cancer after chemotherapy and had significant effects in improving the quality of life, the psychological state, and curative effect of patients. WNNM algorithm had the better noise reduction effect in DWI image processing. This work provided a certain reference for the nursing intervention plan after chemotherapy of early lung cancer.

## 1. Introduction

Lung cancer is a common malignant tumor with high morbidity and mortality, having the significant increasing incidence in the world in recent years [1]. According to the World Health Organization, more than 1.1 million people worldwide die of lung cancer every year, accounting for about 17% of cancer deaths, bringing great pain and economic burden to patients and their families [2]. The clinical characteristics of early lung cancer are not obvious. Most patients have already missed the best period of diagnosis and treatment after clinical symptoms are shown, and the prognosis is extremely poor. Thus, it is easy to relapse and difficult to cure. Medical treatment today is mainly aimed at relieving the clinical symptoms and prolonging life of patients [3]. The main treatment methods for lung cancer include surgical resection, radiotherapy, chemotherapy, and biological therapy. Chemotherapy is the most common treatment method at present, and chemotherapy is combined with other methods for comprehensive treatment in clinical practice [4]. Chemotherapy mainly utilized cytotoxic chemical drugs to remove and kill cancer cells in patients. Although it can relieve the clinical symptoms of patients who cannot receive surgical treatment to a certain extent, its toxic and side effects will cause great damage to the patients' body and mind with the prolongation of chemotherapy period. In particular, the vomiting reaction caused by early chemotherapy affects the patients' quality of life seriously [5, 6]. While killing the cancer cells in the host, it will also reach the whole body with the blood circulation, bringing a series of adverse reactions, such as severe hair loss, nausea, vomiting, and physical weakness [7, 8]. Studies have shown that effective nursing interventions can reduce the discomfort of patients with early chemotherapy [9]. Comfort care is a holistic, creative, and individualized nursing model that enables patients to gain a state of comfort at the psychological, physical, and social levels [10]. Tian et al. [11] studied the effect of comfort care on the rehabilitation quality of patients undergoing oral surgery, and the results showed that comfort care could effectively reduce complications during recovery and deserved a clinical promotion value.

Compared with other imaging examinations, magnetic resonance imaging (MRI) can assess the morphological changes of cancer patients, evaluate the pathological changes of cancer, and provide useful information for the diagnosis and treatment of patients effectively [12]. In the MRI, diffusion-weighted imaging (DWI) is a new imaging technology developed in the middle of the last century. Its working principle is mainly realized by molecular thermal energy stimulation, also known as Brownian motion. At present, this technology has been widely used in the evaluation of chemotherapy effects and prognosis of lung cancer patients [13]. Although DWI can effectively reflect changes in tissue morphology, it still suffers from noise interference during image transmission, which affects the imaging results. With the continuous popularization of artificial intelligence technology, some scholars have used intelligent algorithms to achieve image noise reduction. The weighted nuclear norm minimization (WNNM) algorithm is a low-rank matrix approximation noise reduction algorithm, which is optimized by nuclear norm minimization (NNM). According to the low rank of the image, NNM restores the potential matrix from the noisy image for denoising. However, NNM assigns the same weight to all singular values, which causes them to shrink with the same strength. The WNNM algorithm can assign different weights to different singular values, so the noise reduction effect is significantly improved. Currently, it is widely used in denoising of natural images and medical images [14].

In summary, the prognosis of lung cancer is very poor and there is a risk of recurrence. Chemotherapy is the main clinical treatment for lung cancer currently, but its toxic and side effects can easily cause adverse reactions such as nausea and vomiting, which will affect the quality of life and mental health of patients. Therefore, the DWI noise reduction model under the weighted nuclear norm minimization (WNNM) algorithm for noise reduction was discussed and was applied into comfort care intervention for vomiting management after early chemotherapy and prediction of curative effect. It was expected to provide new strategies for vomiting management after chemotherapy of lung cancer patients.

## 2. Materials and Methods

### 2.1. Research Objects

In this research, 118 patients with lung cancer who were treated at a hospital from February 2020 to February 2022 were chosen as the research objects. The general clinical data of the patients were collected, including the gender, age, and course of the disease. With a random number table method, the patients were divided into the experiment group and the control group, with 59 persons in each group. In the control group, the patients received routine care, while in the experiment group, the patients received comfortable care. This study had been approved by the ethics committee of the hospital, and the patients and their families understand the research situation and signed the informed consent form.

The inclusion criteria are as follows: the general clinical data of the patients were complete; the patients had high compliance; through the clinical diagnosis; and the patients cannot receive surgical treatment. The exclusion criteria are as follows: the patients were suffering from neurological diseases, accompanied by severe cognitive dysfunction; the patients had severe diseases of the heart, lung, liver, kidney, and other organs; the patients had severe blood diseases or infectious diseases; the patients had taken psychotropic drugs recently; the patients were allergic to the drugs needed; and the patients had other malignant tumors.

### 2.2. Nursing Methods

Routine care was given to all patients in the control group, it included basic nursing, health education, psychological care, and diet guidance. Basic nursing required the medical personnel to communicate with the patients in time after admission and assist the patients to be familiar with the hospital and ward environment. After the patients were admitted to the hospital, health education was carried out according to the specific conditions of the patients, mainly including the pathogenesis, clinical manifestations, treatment methods, prognosis, and toxic and side effects caused by the treatment methods. For psychological care, the medical personnel should communicate more with patients, analyze the current psychological issues of patients timely, and answer questions patiently for the patients. In diet guidance, due to the influence of diseases and chemotherapy drugs, the corresponding rules in the diet were formulated for patients. The patients were asked to have a balanced nutrition, drink more water, and eat lightly.

The patients in the experiment group were treated with comfort care, which mainly included environmental care, psychological care, music therapy, diet care, pain care, sleep care, complication care, and posture care. For environmental care, the patients were in a quiet, comfortable, clean, and tidy ward, and staff were arranged for regular cleaning to keep the air fresh, the temperature, humidity, and light suitable in the ward. In terms of psychological care, the medical personnel should actively communicate with patients during their hospitalization and tell them about the pathogenesis, treatment methods, chemotherapy results, possible toxic, side effects, etc. of lung cancer. Health education for patients was regularly conducted, using the successful cases to motivate patients to cooperate with treatment, so as to improve patients' cognition of their own diseases. During treatment, patients were encouraged to join entertaining activities, and professional psychological guidance was provided. For some patients with mental illness, the medical personnel should consult with the family members of the patients to formulate corresponding strategies. As for music therapy, a comfortable environment was created for the patients, to keep the patients have a comfortable position; and some brisk music was played for the patients. In diet care, patients needed adequate nutrition during treatment. The diet plan was made for the patients as the attention was paid to the diversity and richness of the diet. It was advised that the patients should eat more foods rich in vitamins and high protein, and spicy, hard, and greasy diets were contraindicated. Patients with vomiting could be given more digestible vegetables and fruits to promote gastrointestinal motility and reduce vomiting. For sleep care, the daytime sleep should be appropriately reduced, and the temperature, light, and humidity in the ward were adjusted when the patients fell asleep at night. Night treatment should be avoided as much as possible, and external environmental stimulation should be reduced. For some patients who had difficulty in falling asleep, hot bathing, massage, respiratory therapy, etc. could be chosen to help them go to sleep. In the course of treatment, patients were prone to complications such as nausea, vomiting, and bone marrow suppression. The complication care was performed as the infusion rate and medication order were appropriately adjusted. For patients with severe vomiting, antiemetic drugs could be injected as prescribed by the doctor, and oral nursing should be noticed during this period. Posture care could be combined with music therapy. Nursing staff can help the patients choose a proper lying position according to the specific situation after surgery and assist the patients to change the posture and massage the lower limbs regularly.

### 2.3. Imaging Examination

All the patients were examined with a 3.0 T MRI scanner. Before the examination, the breath-holding training was performed on the patients. During the examination, the patients were instructed to lie in a supine position with both upper limbs high, maintained a calm mind, and avoided from coughing during the imaging. The routine examination sequence included T1W1, T2W1, and DWI, and the apparent diffusion coefficient (ADC) maps were obtained in three cases with *b* values of 600 s/mm^2^, 800 s/mm^2^, and 1000s/mm^2^, respectively. The scanning parameters of DWI were set as follows. Time of repetition (TR) was 8000 ms; time of echo (TE) was 85 ms; layer thickness was 5 mm, the interval was 1.0 mm, the matrix was 288 × 224, and the number of excitations (NEX) was 2. Array spatial sensitivity encoding technology (ASSET) was adopted for scanning in a calm breathing state. The scanned data was sent to the ADW4.5 workstation, and Perfusion body tumor software package was used for mapping, analysis, and calculation. Two experienced radiologists evaluated the images, and the final results were those after discussion if there was a disagreement on the images.

### 2.4. WNNM Noise Reduction Algorithm

The WNNM noise reduction algorithm [15] uses the self-similarity of the image to achieve noise reduction, and the self-similarity includes the texture and structure of the image. It was supposed that *n* was an image with noise, *m* was an original image without noise, and *q* was the Gaussian noise variance of *σ*^2^ with a mean value equal to 0. The relationship could be expressed as

(1) $$\begin{array}{c} n=m+q. \end{array}$$

The noise image *n* was divided into multiple small blocks; each small block was represented by *y*_*r*_. Then, the clustering method was used to match similar image blocks in the entire image and stack all similar image blocks to form a matrix *N*_*r*_  with the same characteristics. The relationship was expressed as

(2) $$\begin{array}{c} N_{r}=M_{r}+Q_{r}. \end{array}$$

In equation (2), *M*_*r*_ represented the original image matrix, *Q*_*r*_ represented the Gaussian noise matrix, and *r* represented the *r*th small block. The WNNM noise reduction algorithm realized image noise reduction by assigning different weights to different singular values. Therefore, the algorithm could be used to predict the image block *M*_*r*_ from the matrix *N*_*r*_. Afterwards, the noises in the image were reduced by integrating all the denoised image blocks, and then, the image *m* was obtained. Gaussian noise variance *σ*^2^ was used to normalize the Frobenius norm, so as to obtain the energy function shown in the following equation:

(3) $$\begin{array}{c} M_{r}=\arg\underset{m_{r}}{\min}\frac{1}{\sigma^{2}}{\left\|N_{r}-M_{r}\right\|}_{F}^{2}+{\left\|M_{r}\right\|}_{\omega }. \end{array}$$

*M*_*r*_ was the predicted image block matrix after noise reduction, and ‖*M*_*r*_‖_*ω*_ was the weighted nuclear function matrix, which was expressed as

(4) $$\begin{array}{c} {\left\|M_{r}\right\|}_{\omega }=\underset{\text{t}}{\Sigma }{\left|\omega_{t}\sigma_{t}\left(M_{r}\right)\right|}_{1}. \end{array}$$

In the above equation, *ω*_*t*_*σ*_*t*_(*M*_*r*_) represented the *t*th singular value in the matrix *M*_*r*_, and *ω*_*t*_ was the weight of the *t*th singular value, being expressed as

(5) $$\begin{array}{c} \omega_{t}=\frac{\text{s}\sqrt{\text{p}}}{\left(\sigma_{t}\left(M_{r}\right)+\gamma \right)}. \end{array}$$

In equation (5), *p* referred to the number of similar blocks, *s* was a normal number, and *γ* was a constant to avoid the denominator being 0. However, the singular value in the original image *M*_*r*_  was an unknown number, which was needed to be predicted from the singular value of matrix *N*_*r*_. The calculation could be expressed as

(6) $$\begin{array}{c} {\overset{-}{\sigma }}_{t}\left(M_{r}\right)=\sqrt{\max\left(\sigma_{t}^{2}\left(N_{r}\right)-p\sigma_{p}^{2},0\right)}. \end{array}$$

In equation (6) above, *σ*_*p*_^2^ represented the noise variance of the *p*th similar block, *p* was the number of similar blocks, and *σ*_*t*_^2^(*N*_*r*_) was the *t*th singular value of matrix *N*_*r*_. Thus, $\overset{-}{M_{r}}$ could be predicted. *G*_*ω*_(*Σ*) represented the soft threshold function, which could shrink the singular value and was expressed as

(7) $$\begin{array}{c} G_{\omega }{\left(\Sigma \right)}_{tt}=\max\left(\Sigma_{tt}-\omega_{t},0\right). \end{array}$$

In equation (7), *Σ*_*tt*_ stood for the diagonal element in the singular value matrix *Σ*.

### 2.5. Observation Indicators

The gastrointestinal nausea and vomiting degree standards in the *Common Adverse Events Evaluation Criteria* published by the Department of Health and Human Services of United States [16] were adopted to assess the vomiting of patients before and after treatment. The condition of vomiting was classified into 5 degrees, as shown in Table 1. The Hamilton Depression Scale (HAMD) [17] and Hamilton Anxiety Scale (HAMA) [18] were used to assess the psychological state of patients. The Quality of Life Questionnaire-Core 30 (QLQ-C30) scale [19] was used to assess the quality of life of patients. The electrochemiluminescence method [20] was used to detect serum tumor markers, including neuron-specific enolase (NSE), carbohydrate antigen 19-9 (CA19-9), carcinoembryonic antigen (CEA), and associated antigen of squamous cell carcinoma (SCC).

### 2.6. Statistical Analysis

SPSS20 system was applied for data analysis. The measurement data were expressed in the form of (*x* ± *s*), the independent sample *t*-test analysis was performed for comparison between groups, and the comparison among multiple time periods was performed by analysis of variance with repeatedly measured data. The enumeration data was expressed by percentage (%). In *χ*^2^ test, *P* < 0.05 indicated the difference was of statistical significance.

## 3. Results

### 3.1. Performance Analysis of Algorithms

For exploring the noise reduction effect of the WNNM noise reduction algorithm, the nonlinear diffusion photon mapping (PM) algorithm [21] and the total variation (TV) norm minimization algorithm [22] were introduced. The peak signal-to-noise ratio (PSNR), the structural similarity (SSIM), and the mean square error (MSE) of the three algorithms were compared under 25% Gaussian noise and 50% Gaussian noise, respectively. As shown in Figure 1, when *σ* was 25% Gaussian noise, the PSNR of the WNNM noise reduction algorithm was 112.54 dB, which was higher than that of the PM algorithm (69.87 dB) and the TV algorithm (76.44 dB). The SSIM of the WNNM noise reduction algorithm was 0.99, higher than that of the PM algorithm (0.47) and the TV algorithm (0.69) as well. The MSE of the WNNM noise reduction algorithm was 0.0005, which was lower than that of the PM algorithm (0.0015) and that of the TV algorithm (0.0009). As shown in Figure 2, when *σ* was 50% Gaussian noise, the PSNR of the WNNM noise reduction algorithm was 111.42 dB, higher than that of the PM algorithm (68.77 dB) and that of the TV algorithm (75.92 dB). The SSIM of the WNNM noise reduction algorithm was 0.97, which was higher than those of both the PM algorithm (0.47) and the TV algorithm (0.65). The MSE of the WNNM noise reduction algorithm was 0.0013, which was lower than those of both the PM algorithm (0.0029) and the TV algorithm (0.0024).

### 3.2. Noise Reduction Effect of Three Algorithms

The DWI images of a 63-year-old patient with brain metastases from lung cancer were taken as the example. As shown in Figure 3, the effects of dealing with different noises were compared under three algorithms. It could be observed that under 25% Gaussian noise and 50% Gaussian noise, the image was still fuzzy after noise reduction under the PM algorithm and TV algorithm. The noise reduction effect of the WNNM noise reduction algorithm was the most ideal, and the produced image was clearer, which was conducive to recognition.

### 3.3. Sensitivity, Specificity, and Area under the Curve (AUC) of ADC Map under Different *b* Values

When the *b* value was 600 s/mm^2^, the sensitivity, specificity, and AUC of the ADC map were 0.76, 0.69, and 0.84, respectively. When the *b* value was 800 s/mm^2^, the sensitivity, specificity, and AUC of the ADC map were measured to be 0.95, 0.89, and 0.87, respectively. When the *b* value was 1000 s/mm^2^, the sensitivity, specificity, and AUC of the ADC map were 0.87, 0.89, and 0.83, respectively. The comparative results are shown in Figure 4.

### 3.4. Statistics of General Clinical Data of Patients

In the control group, there were 37 males and 22 females. The average age was 54.32 ± 13.45 years old. 28 patients had an education level of junior high school or below, 17 patients had that of high school or junior college, and 14 patients owned that of a bachelor degree or above. 47 patients had a history of smoking. In the experiment group, there were 34 males and 25 females, with an average age of 56.71 ± 11.05 years old. 24 patients owned a junior high school education level or below, 21 patients had a high school or junior college level, and 14 patients had a bachelor degree or above. 44 patients had a history of smoking. There was no significant difference in general clinical data of patients between the two groups (*P* > 0.05), as more details are shown in Table 2.

### 3.5. Comparison of Vomiting Degrees of Patients after Chemotherapy between the Two Groups

In the experiment group, 27 patients (45.76%) had the vomiting in degree 0 after chemotherapy, 24 patients (40.68%) had that in degree I, 7 patients (11.86%) had that in degree II, 1 patient (1.69%) had that in degree III, and no one was in degree IV. In the control group, 7 (11.86%), 12 (20.34%), 20 (33.90%), 11 (18.64%), and 9 (15.69%) patients had vomiting in degree 0, degree I, degree II, degree III, and degree IV, respectively, after chemotherapy. As shown in Figure 5, the proportion of patients with degree 0 and degree I in the experiment group was higher than that in the control group, and the number of patients in degrees II, degree III, and degree IV was less than that in the control group, showing the differences were statistically significant (*P* < 0.05).

### 3.6. Psychological State Scores of Patients in the Two Groups before and after Nursing

The HAMD scale scores of patients in the control group and the experiment group before care intervention were 38.67 ± 3.05 points and 38.55 ± 2.97 points, respectively. After the care intervention, those in the two groups were 23.52 ± 2.04 points and 16.49 ± 1.2 points, respectively. The scores of the both groups after care intervention were lower than those before the intervention, and the differences were statistically significant (*P* < 0.05). The score of the HAMD scale in the experiment group after care intervention was significantly lower than that in the control group, with the statistically significant difference as well (*P* < 0.05). The HAMA scale scores of patients in the control group and the experiment group before the care intervention were 45.32 ± 2.45 points and 44.78 ± 2.33 points, respectively. The scores in the control group and the experiment group after care intervention were assessed to be 25.98 ± 1.89 points and 17.48 ± 1.37 points, respectively. The HAMA scores of both groups after care intervention were lower than those before the intervention, as the differences were of statistical significance (*P* < 0.05). The HAMA scores in the experiment group after care intervention were significantly lower than those in the control group, with the statistically significant difference (*P* < 0.05). The comparisons of the scores of HAMD and HAMA scales are shown in Figure 6.

### 3.7. The Score on Quality of Life of Patients in the Two Groups

For patients in the control group after care intervention, the physical motor function was scored as 57.22 ± 4.75 points, the social function was scored as 56.85 ± 4.25 points, the pain score was 42.43 ± 3.74 points, and the cognitive function score was 61.2 ± 4.11 points. For patients in the experiment group after care intervention, the physical motor function, social function, pain, and cognitive function were scored to be 89.43 ± 5.42 points, 83.44 ± 4.87 points, 23.71 ± 3.83 points, and 79.86 ± 2.44 points, respectively. The physical motor function score, social function score, and cognitive function score of patients in the experiment group were significantly higher than those in the control group, but the pain score was significantly lower than that in the control group, and the differences were statistically significant (*P* < 0.05).  Figure 7 showed the comparison of the quality of life between two groups.

### 3.8. Levels of Serum Tumor Markers before and after Care Intervention in the Two Groups

After the care intervention, the levels of serum tumor markers of patients in both groups were significantly lower than those before care intervention with the statistically significant differences (*P* < 0.05). After care intervention, the NSE level of patients in the control group was 23.52 ± 1.87 ng/mL, the CEA level was 20.15 ± 1.23 ng/mL, the associated antigen level of SCC was 1.36 ± 0.15 ng/mL, and the CA19-9 level was 96.83 ± 11.33 U/mL. For patients in the experiment group, the level of NSE, CEA, associated antigen of SCC, and CA19-9 was 18.43 ± 1.05 ng/mL, 14.03 ± 1.12 ng/mL, 0.95 ± 0.33 ng/mL, and 64.72 ± 8.45 U/mL, respectively, after care intervention. The levels of serum tumor markers in the experiment group were significantly lower than those in the control group, which was statistically significant (*P* < 0.05), as shown in Figure 8.

### 3.9. Nursing Satisfaction of Patients in Two Groups

In the experiment group, 47 patients were very satisfied, 10 patients were basically satisfied, and 2 patients were dissatisfied. The overall nursing satisfaction was 96.61%, which was significantly higher than that of the control group (81.36%), and the difference was statistically significant (*P* < 0.05). The statistical analysis of the nursing satisfaction is shown in Figure 9.

## 4. Discussion

The incidence of lung cancer is increasing year by year. Chemotherapy is the major clinical treatment method for lung cancer currently. However, due to the side effects of chemotherapy drugs, patients often show nausea and vomiting, hair loss, bone marrow suppression, etc. in varying degrees after chemotherapy [23]. With the development of imaging technology, MRI technology is used to evaluate the process of pathological changes in patients, but the image output process is affected by noise, and the output pictures cannot fully reflect the internal conditions of the lesions in patients [24]. Therefore, the WNNM noise reduction algorithm was utilized to reduce the noise in DWI images and evaluate the treatment and prediction effect of lung cancer after early chemotherapy under comfort care intervention. The PM algorithm and TV algorithm were also introduced and compared with the WNNM noise reduction algorithm. It was found from the results show that, when *σ* was 25% Gaussian noise, the PSNR and SSIM of the WNNM noise reduction algorithm were 112.54 dB and 0.99, respectively, which were higher than those of the other two algorithms. The MSE of the WNNM noise reduction algorithm was obtained as 0.0005, lower than that of the other two algorithms. When *σ* was 50% Gaussian noise, the noise reduction performance of all the three algorithms was decreased, but the WNNM noise reduction algorithm still had good imaging results. In addition to the algorithm discussed, Gurney-Champion et al. [25] proposed a principal component analysis method for model-free denoising of DWI data. Herbst [26] came up with a parallel imaging algorithm that jointly reconstructed all segments of a DWI frame and maintains their phase information, and the effectiveness of the algorithm was proved through experiments. The sensitivity, specificity, and AUC of the ADC map under different *b* values were evaluated. It was suggested that when the *b* value was 800 s/mm^2^, the ADC map had the best sensitivity, specificity, and AUC value of 0.95, 0.89, and 0.87, respectively. It was indicated that the quantitative characteristics of DWI had a certain predictive value for the effect of chemotherapy in patients with lung cancer. Vogl et al. [27] explored the predictive value of ADC in DWI on the response of primary and secondary lung tumor patients undergoing transpulmonary chemical embolism and transarterial chemical perfusion, and the results suggested that the method was of great value in diagnosis and treatment.

In this research, patients in the control group with routine care and those in the experiment group with comfort care were comprehensively evaluated through experiments. The results showed that the incidence of vomiting in the experiment group was significantly lower than that in the control group with a statistically significant difference (*P* < 0.05), showing the comfort care gave a better effect in improving vomiting in chemotherapy patients. This was because comfort care improved the comfort level of patients during treatment to a certain extent, made patients keep a comfortable state, and relieved the discomfort of lung cancer patients during chemotherapy to the greatest extent [28]. Not only the physical comfort but also the psychological comfort was taken into consideration. After care intervention, the scores of the HAMD scale and HAMA scale of patients in the experiment group were 16.49 ± 1.2 points and 17.48 ± 1.37 points, respectively, which were significantly lower than those of patients in the control group with differences statistically significant (*P* < 0.05). Psychological care was one of the important items in the comfort care. Guiding patients to maintain a good attitude towards the disease could alleviate the anxiety and depression of the patients effectively, and it was of great significance for improving the degree of cooperation between medical personnel and patients. In the quality of life, the scores of physical motor function, social function, and cognitive function of patients in the experiment group were higher than those in the control group, and the pain score was lower than that in the control group (*P* < 0.05). It was observed that comfort care had a significant effect in improving the quality of life of patients. The reason was that the process of comfort care required health education and psychological care for patients, and patients were helped to develop good living habits. Thereby, the confidence and compliance of patients were enhanced in the treatment of diseases, guaranteeing the curative effect effectively [29]. From the results of the serum tumor marker levels, the level of NSE, CEA, associated antigen of SCC, and CA19-9 of patients in the experiment group was 18.43 ± 1.05 ng/mL, 14.03 ± 1.12 ng/mL, 0.95 ± 0.33 ng/mL, and 64.72 ± 8.45 U/mL, respectively, which was significantly lower than those in the control group (*P* < 0.05). CA19-9 is a tumor-associated antigen, CEA is the carcinoembryonic antigen, and the associated antigen of SCC is a glycoprotein subtype of tumor-associated antigen. The serum levels of these three substances will increase in patients with lung cancer. NSE is one of the enolases involved in glycolytic pathway, and it is mostly found in neuroendocrine tissues; its serum level in patients is often used as a clinical diagnostic indicator [30]. The serum levels of four serum tumor markers in patients in the experiment group were significantly lower than those in the control group, indicating that the effect of comfort care treatment was better. Finally, the nursing satisfactions of patients were compared between the two groups. The results suggested that the overall nursing satisfaction of the experiment group was 96.61%, higher than that of the control group significantly (*P* < 0.05). It could be observed that comfort care had a better effect on improving the nurse-patient relationship and improving nursing satisfaction of patients.

## 5. Conclusion

Examination was performed by WNNM-based DWI in the control group with routine care and the experiment group with comfort care. The relevant clinical indicators were also evaluated comprehensively. The DWI images optimized by the WNNM algorithm were clear with less noise, which was beneficial to clinical diagnosis and had a certain predictive function on the chemotherapy effect of lung cancer patients. Comfort care could relieve the vomiting reaction effectively of patients with lung cancer chemotherapy, showing notable effects in improving the quality of life, psychological state, and curative effect of patients. The deficiencies of this research lay in the lacks of comparative analysis of DWI and other imaging methods as well as the research results of a large sample size. Future research is needed to discuss the long-term impact of comfort care. This work provided data support for the formulation of nursing programs for lung cancer patients undergoing chemotherapy.

## Figures and Tables

**Figure 1:** Evaluation of noise reduction performance of three algorithms when *σ* was 25% Gaussian noise. (a–c) Show the comparisons of PSNR, SSIM, and MSE, respectively.

**Figure 2:** Evaluation of noise reduction performance of three algorithms when *σ* was 50% Gaussian noise. (a–c) Show the results of PSNR, SSIM, and MSE, respectively.

**Figure 3:** The noise reduction effect of the three algorithms under different Gaussian noises. (a, e) Are the original images with Gaussian noise; (b, f) are the images processed by PM algorithm; (c, g) are those denoised by the TV algorithm; (d, h) are those obtained by the WNNM noise reduction algorithm.

**Figure 4:** Sensitivity, specificity, and AUC of ADC map under different *b* values. (a–c) Show the comparison of the sensitivity, specificity, and AUC, respectively.

**Figure 5:** Comparison of vomiting degrees of patients between the two groups after chemotherapy. (a) Shows the population statistics, while (b) shows the constituent ratio. ^∗^Compared with those in the experiment group, *P* < 0.05.

**Figure 6:** Scores on the psychological state of patients in the two groups before and after care intervention. (a, b) Show the scores of HAMD and HAMA scales, respectively. ^∗^Compared to the scores in the experiment group; ^#^compared to those after care intervention, *P* < 0.05.

**Figure 7:** Quality of life scores of patients in the two groups. ^∗^Compared with experiment group, *P* < 0.05.

**Figure 8:** Comparison of serum tumor markers' levels of patients before and after care intervention between the two groups. (a–d) Show the comparisons of NSE, CEA, associated antigen of SCC, and CA19-9, respectively. ^∗^Compared with experiment group; ^#^compared with those after care intervention, *P* < 0.05.

**Figure 9:** Nursing satisfaction of patients in the two groups. ^∗^Compared to the satisfaction of the experiment group, *P* < 0.05.

**Table 1:** Degrees of vomiting.

Degrees	Explanations
Degree 0	The patients had no vomiting in the day.
Degree I	The patients vomited once a day, which was mild nausea.
Degree II	The patients vomited 2 to 5 times a day, which was temporary nausea and vomiting.
Degree III	The patients vomited more than 6 times a day and needed parenteral nutrition and intravenous fluids for recovery.
Degree IV	The patients had severe vomiting, which still cannot be relieved after drug control.

**Table 2:** Statistics of general clinical data of patients.

Items		Control group (*n* = 59)	Experiment group (*n* = 59)
Gender	Male (*n*)	37	34
	Female (*n*)	22	25
Age (years old)		54.32 ± 13.45	56.71 ± 11.05
Education level	Junior high school or below (*n*)	28	24
	High school or junior college (*n*)	17	21
	Bachelor degree or above (*n*)	14	14
History of smoking	Smokers (*n*)	47	44
	Nonsmoker (*n*)	12	15

## Data Availability

The data used to support the findings of this study are available from the corresponding author upon request.
